# Construction of circRNA-Associated ceRNA Network Reveals Novel Biomarkers for Esophageal Cancer

**DOI:** 10.1155/2020/7958362

**Published:** 2020-08-28

**Authors:** Yunhao Sun, Limin Qiu, Jinjin Chen, Yao Wang, Jun Qian, Lirong Huang, Haitao Ma

**Affiliations:** ^1^Department of Thoracic Surgery, The First Affiliated Hospital of Soochow University, China; ^2^Department of Thoracic Surgery, Yancheng City No.1 People's Hospital, China; ^3^Oncology Department, Yancheng City No.1 People's Hospital, China

## Abstract

**Objective:**

Esophageal cancer (ESCC) is reported to be the eighth most common malignant tumors worldwide with high mortality. However, the functions of majority circRNAs in ESCC requires to be further explored.

**Methods:**

This study identified differently expressed circRNAs in 3 paired ESCC using RNA-sequencing method. The interactions among circRNAs, miRNAs, and mRNAs were predicted using bioinformatics analysis.

**Results:**

In this study, using RNA-sequencing method and integrated bioinformatics analysis, 418 overexpressed circRNAs and 637 reduced circRNAs in ESCC sample were identified. Based on the mechanism that circRNAs could play as ceRNAs to modulate targets expression, circRNA-miRNA and circRNA-miRNA-mRNA networks were constructed in this study. Based on the network analysis, 7 circRNAs, including circ_0002255, circ_0000530, circ_0001904, circ_0001005, circ_0000513, circ_0000075, and circ_0001121, were identified as key circRNAs in ESCC. We found that circ_0002255 was related to the regulation of substrate adhesion-dependent cell spreading. circ_0001121 was involved in regulating nucleocytoplasmic transport. circ_0000513 played a key role in regulating Adherens junction, B cell receptor signaling pathway. Meanwhile, we observed circ_0000075 was involved in regulating zinc II ion transport, transition metal ion homeostasis, and angiogenesis.

**Conclusion:**

We thought this study could provide novel biomarkers for the prognosis of ESCC.

## 1. Introduction

In recent years, the functional importance of noncoding RNAs (ncRNAs) in the tumorigenesis and the development of cancers have been found. CircRNAs are a type of special endogenous RNA molecules [1]. With the development of high-throughput RNA sequencing, circRNAs were found to be present in human cells. Emerging reports have revealed the important roles of circRNAs in multiple human diseases, such as malignant tumors [1–3]. The findings indicated that circRNAs were abnormally expressed and involved in regulating cancer proliferation and therapy resistance through various mechanisms, such as sponging miRNAs or proteins, and regulating RNA splicing and transcription [3–5].

Esophageal cancer (ESCC) is reported to be the eighth most common malignant tumors worldwide with high mortality [6, 7]. Previous studies showed more than 455800 patients were diagnosed with ESCC, and almost 400200 patients died from this disease [8]. Despite novel methods, such as radiotherapy and chemotherapy, were used in the ESCC treatment, the five-year survival rate of ESCC patients is as low as about 25% due to distant metastasis and therapy resistance [9, 10]. It is therefore of great importance to explore an effective treatment to prevent ESCC progression.

A number of reports have indicated that circRNAs were related to the development of ESCC. A report by Chen et al. showed circLARP4 suppressed ESCC progression via sponging miR-1323 and modulating PI3K signaling [11]. Another study by Pan et al. found that hsa_circ_0006948 modulated miR-490-3p/HMGA2 axis, thus regulating tumorigenesis and EMT processes in ESCC [12]. Moreover, the special expression pattern of circRNAs in ESCC was validated as potential biomarkers for the prognosis of this disease. For example, hsa_circRNA_100873 upregulation was correlated to lymphatic metastasis of ESCC [13], and Circ-SLC7A5 was validated as a potential prognostic circulating biomarker for detection of ESCC, which was correlated to advanced stage and worse prognosis [14]. Despite a few studies revealed the functions of circRNAs in ESCC [15, 16], the functions of majority circRNAs require to be further explored.

Recently, the progress in RNA-sequencing method had expanded the understanding of the molecular mechanism of cancers. A series of novel mRNAs and noncoding RNAs were revealed to be related to the tumorigenesis. For example, Li et al. revealed that circDDX17 was downregulated in colorectal cancer with RNA sequencing and suppressed tumor development [17]. Huang et al. reported abundant mRNA, circRNA, and lncRNA in blood could act as diagnostic markers for cancers by using extracellular vesicles long RNA sequencing [18]. Yu et al. found hsa_circ_0001445 was identified to be downregulated by RNA-sequencing and suppress liver cancer metastasis [19]. Also, using RNA-sequencing method could provide novel biomarkers for ESCC.

This study identified differently expressed circRNAs in ESCC using RNA-sequencing method. The interactions among circRNAs, miRNAs, and mRNAs were predicted using bioinformatics analysis. We thought this study was able to provide novel biomarkers for ESCC.

## 2. Materials and Methods

### 2.1. Tissue Specimens

Three paired ESCC tissues and adjacent normal tissues were collected from patients who received radical gastrectomy at the Department of Thoracic Surgery, The First Affiliated Hospital of Soochow University, from 2019 to 2020. All specimens were collected under the guidance of the HIPAA protocol and supervised by the ethics committee. TNM stage classification complied with the TNM classification system of the International Union Against Cancer (7th edition). These patients were diagnosed with ESCC with average age: 62.7.

### 2.2. RNA-seq Analysis

The total RNA was isolated with RNAiso Plus (TaKaRa Japan). The Ribo-Zero rRNA Removal Kit (Illumina, San Diego, CA, USA) and the CircRNA Enrichment Kit (Cloud-seq, USA) were used to remove the rRNA and enrich the circRNAs. The RNA-seq libraries were constructed by using TruSeq Stranded Total RNA Library Prep Kit (Illumina, San Diego, CA, USA). The libraries were denatured as single-stranded DNA molecules, captured on Illumina flow cells, amplified in situ as clusters, and finally sequenced for 150 cycles on Illumina HiSeq™ 4000 Sequencer (Illumina, San Diego, CA, USA). All these assays were conducted according to the manufacturer's instructions. The raw data were listed as a supplementary table 1.

### 2.3. Identification and Quantification of Human circRNAs

For each sample, the cleaned RNA-seq reads were first mapped to the human reference genome (GRCh37/hg19, UCSC Genome Browser [20]) by TopHat2 [21]. Then, the unmapped reads of each sample in the TopHat2 results were used to identify the circRNAs by UROBORUS pipeline [22].

### 2.4. Differential Expression Analysis

Differentially expressed circRNAs between ESCC and normal samples were determined using the “limma” package (3.38.3) in R (5.3.2) [23, 24]. A paired Student's *t*-test was used to identify any significant differences in circRNA expression between tumor and tumor-adjacent normal tissues. The thresholds of foldchange >2 were set to screen the significantly DESCCs.

### 2.5. Functional Analysis

Bioinformatics analysis was conducted using the DAVID online database (https://david.ncifcrf.gov/home.jsp) [25]. The results were visualized by the imageGP online software (http://www.ehbio.com/ImageGP/index.php/Home/Index/index.html).

### 2.6. Correlation Analysis of circRNAs and mRNAs in ESCC

An Agilent circRNA and mRNA expression profile microarray was used to screen the differentially expressed circRNA and mRNA gene expression. The regulation of the mRNA target expression of circRNAs was evaluated to investigate whether circRNAs could act as “miRNA sponges.” CircRNA-miRNA interaction analysis was conducted by Cytoscape 3.2.1 software (Cytoscape Consortium). The size of each node represents the number of putative miRNAs that were functionally connected to each circRNA.

## 3. Result

### 3.1. Identification and Validation of Differentially Expressed circRNAs in ESCC

By analyzing the expression pattern of circRNAs between ESCC tumors and normal tissues, 1055 circRNAs were identified to be differently expressed in ESCC tissues with fold change ≥2 (Figures 1(a) and 1(b)). Among these circRNAs, 418 circRNAs were overexpressed, and 637 circRNAs were reduced in ESCC sample compared to normal tissues (Figure 1(c)). Heatmap and volcano plot analysis demonstrated these significant differentially expressed circRNAs (Figures 1(a) and 1(b)).

### 3.2. Enrichment Analysis of circRNAs' Parental Genes

Furthermore, we perform GO analysis to explore the potential functional roles of circRNAs' parental genes. Our results showed that the top 10 biological processes related to parental genes of differently expressed circRNA included cellular component organization, biosynthetic process, macromolecule biosynthetic process, primary metabolic process, RNA metabolic process, and transcription from RNA polymerase II promoter (Figure 2(a)). Meanwhile, the top 10 molecular functions and cellular components related to these circRNAs' parental genes were shown in Figures 2(b) and 2(c).

The KEGG analysis revealed that the pathways related to parental genes of differently expressed circRNAs included ErbB signaling pathway, focal adhesion, and lysine degradation (Figure 2(d)).

### 3.3. Construction of circRNA-miRNA-mRNA Network

A number of studies showed circRNAs act as sponges of miRNA to suppress their activities. Therefore, we constructed a circRNA-miRNA interaction network using bioinformatics methods. The interaction between circRNA and miRNAs was predicted using circinteractome database (https://circinteractome.nia.nih.gov/) [26].

Next, we constructed a circRNA-miRNA-mRNA network in ESCC. The miRNA-mRNA pairs were identified using Starbase [27] and TARGETSCAN [28] database. A total of 8975 mRNAs were identified as potential circRNA-miRNA targets. Then, we extracted differently expressed mRNAs in ESCC using GEPIA database [29]. Finally, ESCC specific circRNA associated ceRNA network was constructed with Cytoscape 3.6.1 software [30], which included 7 circRNAs (circ_0002255, circ_0000530, circ_0001904, circ_0001005, circ_0000513, circ_0000075, circ_0001121), 7 miRNAs (hsa-miR-31-5p, hsa-let-7i-5p, hsa-miR-4644, hsa-miR-105-5p, hsa-miR-370-3p, hsa-miR-544a, hsa-miR-17-3p), and 548 mRNAs (Figures 3(a) and 3(b)).

### 3.4. Enrichment Analysis of Key circRNAs in This Network

Next, we conducted the bioinformatics analysis of Key circRNAs in this network using Clue-GO plugin [31] in Cytoscape 3.6.1 software. The results revealed that hsa_circ_0002255 was related to the regulation of substrate adhesion-dependent cell spreading (Figure 4(a)). hsa_circ_0001121 was involved in regulating nucleocytoplasmic transport and protein export from nucleus (Figure 4(b)).

Moreover, we identified hsa_circ_0000513 played a key role in regulating Adherens junction, B cell receptor pathway, ERBB signaling, pri-miRNA transcription, regulation of phosphatase activity, histone phosphorylation, and protein processing in endoplasmic reticulum (Figure 4(c)). Among these pathways, we specially indicated that ERBB signaling was potentially regulated by this circRNA via PTPRJ, SOS1, HIP1, PXN, and PIGU.

Meanwhile, we observed hsa_circ_0000075 was involved in regulating zinc II ion transport, transition metal ion homeostasis, angiogenesis, blood vessel development, extrinsic apoptotic signaling pathway, response to amino acid, nucleocytoplasmic transport, response to acid chemical, toll-like receptor 4, cellular response to hepatocyte growth factor stimulus, chemotaxis transforming, and growth factor beta2 production (Figure 4(d)).

### 3.5. The Dysregulation of Key miRNAs Was Related to the Survival Time in ESCC

Next, we predicted the prognostic value of key miRNAs in ESCC with TCGA data. The results showed that higher expression level of hsa−let−7i (Figure 5(a)), hsa−mir−4644 (Figure 5(b)), hsa−mir−17 (Figure 5(c)), hsa−mir−544a (Figure 5(d)), hsa−mir−105 (Figure 5(e)) were associated with shorter overall survival time in ESCC patients.

## 4. Discussion

Recently, the circRNAs have been reported to be related to ESCC. CircRNA dysregulation was related to prognosis and tumor proliferation regulation of ESCC. For example, Zhang et al. revealed 2,046 circRNAs were frequently altered in ESCC tissues [32]. Su et al. identified 57 induced circRNAs and 17 reduced circRNAs in radioresistant ESCC cells compared to normal ESCC cells [33]. Also, the special functions of several circRNAs had been clearly demonstrated. For example, CiRS-7 promotes growth and metastasis of ESCC via regulation of miR-7/HOXB13 [34]. However, these studies just revealed a limited amount of circRNAs in ESCC. According to circBase database, more than 50000 circRNAs exited in human cells [35]. Therefore, this was still an urgent need to identify differently expressed circRNAs in ESCC to expand our understanding of the mechanism related to ESCC development. In this study, using RNA-sequencing method and integrated bioinformatics analysis, 418 overexpressed circRNAs and 637 reduced circRNAs in ESCC sample were identified. Based on the mechanism that circRNAs could play as ceRNAs to modulate targets expression [36, 37], circRNA-miRNA and circRNA-miRNA-mRNA networks were constructed in this study. Based on the network analysis, 7 circRNAs, including circ_0002255, circ_0000530, circ_0001904, circ_0001005, circ_0000513, circ_0000075, and circ_0001121, were identified as key circRNAs in ESCC. We found that circ_0002255 was related to the regulation of substrate adhesion-dependent cell spreading. circ_0001121 was involved in regulating nucleocytoplasmic transport. circ_0000513 played a key role in regulating Adherens junction, B cell receptor signaling pathway. Meanwhile, we observed circ_0000075 was involved in regulating zinc II ion transport, transition metal ion homeostasis, and angiogenesis.

CircRNAs have been shown to function as regulators of parental gene transcription and alternative splicing and miRNA sponges. Exon–intron circular RNAs (EIciRNAs) hold U1 snRNP through interaction with U1 snRNA, and then, the EIciRNA–U1 snRNP complexes further interact with Pol II transcription complex at the promoters of parental genes to enhance gene transcription and expression [38, 39]. Zhang et al. [39, 40] found that circEIF3J and circPAIP2 with higher expression levels can complement U1 and interact with U1 small ribonucleoprotein to promote the transcription of EIF3J and PAIP2 genes in cis. Intronic circRNAs (CiRNAs) also positively regulate Pol II transcription. For example, ci-ankrd52, generated from gene ANKRD52, is capable of accumulating to its transcription sites and regulates elongation Pol II machinery acting as a positive regulator for transcription [39]. Moreover, circRNAs could acted as ceRNAs to affect parental gene expression. For example, circ-VANGL1 as a competing endogenous RNA modulates VANGL1 expression via miR-605-3p [41]. Thus, prediction of the molecular functions related to circRNAs' parental genes could provide more clues to understand the potential functions of circRNAs. The present study showed the pathways related to parental genes of differently expressed circRNAs included ErbB signaling pathway, focal adhesion, and lysine degradation.

Recently, circRNA-mediated ceRNA pathways played a crucial role in cancer initiation and development. For example, circRNA-UCK2 suppressed prostate cancer viability and metastasis through sponging miRNA-767-5p [42]. circFOXO3 was found to promote prostate cancer and glioma progression through sponging miR-29a-3p [43] and miR-138-5p [44]. CircPTPRA suppressed bladder cancer via sponging miR-636 [45]. Also, several cancer-related ceRNA networks were identified. Song et al. constructed a colorectal cancer-related ceRNA network, which includes 13 circRNAs, 62 miRNAs, and 301 mRNAs [46]. In this study, we for the first time built a miRNA-mRNA network in ESCC, containing 33 circRNAs and 158 miRNAs. hsa_circ_0001904, hsa-miR-1273g-3p, hsa-miR-6089, hsa-miR-6873-3p, hsa-miR-8485, and hsa-miR-939-5p were identified as key regulators in ESCC. miR-1273g was found to suppress colorectal cancer proliferation via activation of AMPK signaling [47]. hsa-miR-6089 played a crucial role in regulating inflammation through regulating TLR4 [48, 49]. miR-939 had been revealed to be a key regulator in human cancers, including lung cancer [50], colorectal cancer [51], tongue squamous cell carcinoma [52], epithelial ovarian cancer [53, 54], and gastric cancer [55]. Overexpression of this miRNA enhanced lung cancer progression [50]. In gastric cancer, knockdown of miR-939 modulated metastasis and chemoresistance via dysregulation of SLC34A2 and Raf/MEK/ERK pathway [55].

Also, we built an ESCC-related circRNA-miRNA-mRNA network, including 7 circRNAs, 7 miRNAs, and 548 mRNAs. Very interestingly, bioinformatics analysis showed that hsa_circ_0000513 played a key role in regulating ERBB signaling pathway, regulation of pri-miRNA transcription, and histone phosphorylation in endoplasmic reticulum. ERBB signaling pathway was reported to be activated in ESCC [56, 57]. For example, inhibitors of ERBB signaling were found to suppress ESCC cell migration. miRNAs played an important role in ESCC via affecting cell growth, migration, and autophagy. Very interestingly, we showed hsa_circ_0000513 may affect miRNA functions through modulating their transcription. A recent study showed hsa_circ_0000075 participated in the AF pathogenesis via TGF-beta signaling pathway. However, the roles of hsa_circ_0000075 in ESCC remained unclear. The present study showed that hsa_circ_0000075 was involved in regulating angiogenesis, blood vessel development, and regulation of extrinsic apoptotic signaling pathway.

Despite this study identified differently expressed circRNAs and predicted their functions in ESCC with bioinformatics method, several limitations should be noted. Firstly, the molecular functions and mechanisms of these circRNAs should be further confirmed using experimental assays. Secondly, the prognostic value of key circRNAs should be further explored. The correlation between circRNAs expression and tumor stage, survival time should be further evaluated with collected clinical samples. Finally, the raw data of the Ribo-zero library-based RNA-seq data should be further analyzed to confirm circRNA-mRNA interaction in the future study.

In our study, we identified 418 overexpressed circRNAs and 637 downregulated circRNAs in ESCC and conducted bioinformatics to reveal the potential mechanisms and molecular functions of these circRNAs in ESCC. We thought this study could provide novel biomarkers for the prognosis of ESCC.

## Figures and Tables

**Figure 1:** Analysis of differentially expressed circRNAs in ESCC by RNA-sequencing. (a) Heatmap analysis of differentially expressed circRNAs between ESCC and normal groups. (b) The volcano plot analysis of differentially expressed circRNAs between ESCC and normal groups. (c) The summarization of upregulated and downregulated circRNAs between ESCC and normal groups.

**Figure 2:** In silico analysis of circRNAs' parental genes. (a) Enrichment of the top 10 BP of circRNAs' parental genes. (b) Enrichment of the top 10 MF of circRNAs' parental genes. (c) Enrichment of the top 10 CC of circRNAs' parental genes. (d) Enrichment of the top 10 pathways of circRNAs' parental genes. The size: the number of genes. MF: molecular functions; CC: cellular components; BP: biological processes.

**Figure 3:** Construction of circRNA associated ceRNA network. Green circle: upregulated circRNAs; red circle: downregulated circRNAs; blue circle: miRNAs; purple circle: upregulated mRNAs; deep blue circle: downregulated mRNAs.

**Figure 4:** Enrichment analysis of key circRNAs. (a) Enrichment of hsa_circ_0002255 in esophageal cancer. (b) Enrichment of hsa_circ_0001121 in esophageal cancer. (c) Enrichment of hsa_circ_0000513 in esophageal cancer. (d) Enrichment of hsa_circ_0000075 in esophageal cancer. The circle: biological pathways; the dots: genes.

**Figure 5:** The dysregulation of key miRNAs was related to the survival time in ESCC (a–e) higher expression level of hsa−let−7i (a), hsa−mir−4644 (b), hsa−mir−17 (c), hsa−mir−544a (d), hsa−mir−105 (e) were associated with shorter overall survival time in ESCC patients.

## Data Availability

The data used to support the findings of this study are available from the corresponding author upon request.

## Supplementary Materials

Supplementary Materials Supplementary Table 1: the different expressed circRNAs in ESCC.
